The article "Characteristics of COVID-19 and Research Progresses on Genetic Engineering Vaccine Based on Big Data" was published in 2022. Journal: J Healthc Eng.

# Characteristics of COVID-19 and Research Progresses on Genetic Engineering Vaccine Based on Big Data

**DOI:** 10.1155/2022/9311052

**Published:** 2022-02-26

**Authors:** Qixing Wei

**Affiliations:** Biotechnology Department, Beijing University of Chemical Technology, Beijing, China

## Abstract

Big data platforms can effectively analyze the data and maximize the value of the data by mining the text, digital, video, and image data in various industries. The combination of big data and various industries has brought great changes to the development of the industry. Providing data according to demand can save more time and promote the development of the industry. SARS-CoV-2 (COVID-19) is sweeping across the world, and it has spread to several countries and regions. Human infections have been reported all around the world. Due to the unique characteristics of COVID-19, no specific medicine is available yet to cure patients before the successful research and development of vaccines. Hence, it is of important significance to research and develop vaccines. Guided by the biological characteristics of COVID-19 and the philosophy of synthetic biology, this study reviews the developed genetic engineering vaccines.

## 1. Background

In November 2019, patients with novel coronavirus pneumonia (COVID-19) were identified in Wuhan, and subsequently, patients with COVID-19 were reported in many provinces in China and abroad. As of March 2020, the World Health Organization (WHO) declared a global pandemic of coronavirus disease 2019, and many countries adopted strict blockade measures. As of June 2020, the number of patients with COVID-19 is close to 8 million.

According to clinical data, COVID-19 is initially asymptomatic, and patients with positive nucleic acid tests have no early fever. Some patients have early temperature fluctuations between 36.5°C and 38°C, but the body temperature is lower than 39°C [1]. Studies have shown that even patients without overt symptoms have an extremely high capacity for virus transmission. Only a small number of mildly ill patients show extensive infection shadows on lung CT after hospitalization, and most patients have good lung findings. However, RNA of COVID-19 was found in the laryngeal tissue of both severely and mildly ill patients.

COVID-19 belongs to the RNA viruses and contains four main structural proteins, namely, the macrospin (S glycoprotein), which forms a polymer, the *M* glycoprotein, which wraps the RNA and internal proteins, and the phosphorylated N and E proteins [2]. Outbreak viruses belong to beta-coronaviruses. *β*-coronaviruses with similar fragments have been identified in bats through evolutionary trees. Therefore, it is presumed that the main transmission route of COVID-19 is associated with bats.

Vaccines are known to be the simplest and most direct means of stopping epidemics. However, because COVID-19 is so strongly mutated, it is difficult to develop a vaccine. Currently, vaccine development is mainly based on the structural features of the viral S protein. The S protein mediates the binding of the virus to the host cell and becomes the key to vaccine development. Currently, there are many bioinformatics methods used for vaccine structure design. Since the infection characteristics of COVID-19 are similar to those of historical SARS and MERS, this study provides a comparative analysis of these three viruses with the aim of gaining experience in the development of specific vaccines.

## 2. Relations of COVID-19 with SARS and MERS

It is essential to study the relationship of new coronaviruses with other coronaviruses in human history. By analyzing previous viruses and their relationship to COVID-19, vaccine development can be made less difficult and shorter. Severe acute respiratory syndrome (SARS) and Middle East respiratory syndrome (MERS) are two coronavirus outbreaks associated with COVID-19. SARS was an outbreak 17 years ago and has a high structural similarity to COVID-19 and is, therefore, closely related. Middle East respiratory syndrome is the most recent coronavirus outbreak prior to COVID-19. Based on the abovementioned understanding, it is tentatively suggested that COVID-19 may have some connection with MERS and SARS. By analyzing the similarities between the new coronavirus vaccine and MERS and SARS, it will facilitate researchers to further determine the direction of the new coronavirus vaccine development.

The structural proteins of viruses are the key to determine the type of virus. Therefore, determining the relationship between these viruses must start from the similarities and differences of the related structural proteins. First, the genes encoding the structural proteins of the viruses need to be analyzed, and the degree of gene sequence similarity can generally help researchers determine their relationship to COVID-19.

Although the timing of MERS was closest to the outbreak of COVID-19, the structural protein gene sequences of COVID-19 were more than 90% similar to those of SARS. Based on bioinformatics analysis, COVID-19 is closer to SARS in the evolutionary tree. Therefore, studying the available SARS data can yield more background data related to COVID-19 [3]. Since the S and N proteins of viruses are usually conserved, vaccines prepared based on the structure of S and N proteins in viruses have a long validity period.

## 3. ACE2 Is the Receptor of COVID-19 Cells

By analyzing the S proteins in SARS and COVID-19, scientists found 76% similarity between the S proteins of the two viruses, implying that similar proteins on cells may be used as receptors to enter cells when SARS and COVID-19 invade them. ACE2 is an important channel for SARS viruses, while SARS-CoV S-MLV and SARS-CoV-2 S-MLV have the same ability to enter cells. In this experiment, ACE2 was found to be a receptor for multiple coronaviruses to enter cells. Based on further sequence analysis of the SARS glycoprotein, ACE2 is a receptor for COVID-19, which binds to COVID-19 and mediates its entry into cells [4].

Subsequently, the cellular infection behavior of COVID-19 was analyzed. Similarly, cellular infection by SARS was used in the comparative analysis. The researchers analyzed the similarities and differences between SARS and COVID-19 based on the way they bind to ACE2. According to previous studies, the glycoprotein of SARS has 14 key binding sites to ACE2. However, the analysis of COVID-19 binding to ACE2 revealed that 8 of the 14 sites were extremely conserved and the remaining 6 were semiconserved sites. This study explains the similarity of SARS and COVID-19 [4].

Based on the abovementioned analysis, scientists used cryoelectron microscopy to observe the specific binding sites of S proteins to ACE2. By observing the trimmers formed by S proteins (S1 subunit and S2 subunit) with ACE2, it was found that the glycoprotein S2 subunit binds to the ACE2 protein in a very similar form in both viruses.

## 4. Epitopes on T Cells and B Cells

Under all conditions, the targets recognized by t cells are peptide fragments derived from exogenous proteins. These peptide fragments are captured by specific molecules of the host cell and presented to the cell surface. The molecules that submit antigenic peptides to t cells are cell membrane glycoproteins encoded by a complex set of major histocompatibility complex (MHC) genes. Researchers can design experiments to study the response of t cells and b cells to a given antigen. It has been reported that 27 of 115 epitopes on the surface of t cells are involved in COVID-19 responses, all of which target the S and N proteins of COVID-19 [5]. However, very few of them are able to produce their neocoronavirus counterpart genes. Similar to t cells, b cells have some epitopes that produce binding responses to the structural proteins of COVID-19. Although only some individuals possess MHC genes capable of producing responses to COVID-19 structural proteins, generating epitopes for binding responses is essential for vaccine [4] studies. Immune cells can respond to the structural protein of COVID-19, thus helping researchers to discover the binding sites of COVID-19 structural protein. Different epitopes on immune cells can generate coupling reactions with different structural proteins on COVID-19, which facilitates researchers to identify the binding sites of COVID-19 [6] structural proteins. By integrating the coupling reactions, the true key proteins can be screened from the many binding sites of the structural proteins, thus screening the most critical protein subassociations that recognize COVID-19. By analyzing the sequence and spatial structure of the key proteins and their subconjugation, a COVID-19 vaccine can be further developed.

## 5. An Effective Vaccine Is Needed to Resist COVID-19

There are no specific anti-neocoronavirus drugs available, and all patients who are cured have the virus killed in their bodies through medical care and autoimmunity. Therefore, there is a need to develop a vaccine to stop the further spread of the new coronavirus. Vaccination of the public develops general immunity to the new coronavirus and weakens the ability of COVID-19 to infect and spread. Currently, many countries around the world are giving sufficient attention to vaccine development. Many companies related to the medical industry around the world are investing a lot of manpower and capital in the development of new coronavirus vaccines. According to incomplete statistics, pharmaceutical companies are working on five main technological lines, including the development of inactivated vaccines, recombinant protein vaccines, nucleic acid vaccines, adenovirus vector vaccines, and attenuated influenza virus vaccines.

The research and development of laboratory vaccines is based on the infectious behavior of the virus. That is, virus samples need to be obtained before a vaccine can be studied, but in practice, the virus is generally not collected directly from patients. It is claimed that the operation of collecting virus directly from patients is very complex. The limitations of the direct sampling method are even more pronounced when the laboratory is far from the infected area. For example, it may lead to virus leakage. Therefore, the traditional method of studying viruses in the laboratory is to query the genetic sequence of the virus through international databases (e.g., NCBI) and then synthesize a clone of the currently prevalent virus artificially in the laboratory. Finally, clones are used as the basis for research.

In the early stages of a viral plague outbreak, research teams are often organized in the country of origin to investigate the infected individuals. Several suspected pathogens are extracted from the patients. Later, each of these suspected pathogens is analyzed according to Koch's law and the pathogen of the outbreak is finally identified. The viral pathogen required structural analysis and genetic sequence analysis to determine the virus type and to publish the genetic sequence of the virus to the world. Later, research departments around the world used the published gene sequences as the basis for studying the virus by various means.

When a virus is synthesized in the laboratory, a reverse genetics approach must be used. In other words, we must understand the specific functions of different genes in the context of known viral gene sequences. Synthetic viruses are synthesized in engineered bacteria. The cDNA of the virus must be obtained, since the virus is synthesized in engineered bacteria. The cDNA of the virus is fed into a recombinant plasmid, which is then fed into the engineered bacterium. Finally, the virus is assembled in the engineered bacterium [7].

In the plasmid expression system, the cDNA of the virus is inserted into the gap between the RNA polymerase I promoter and terminator. At the same time, the entire transcription unit of RNA polymerase I is surrounded by the promoter and terminator of RNA polymerase II. This structure is known as the polii-polii structure. In this structure, the expression of RNA polymerase I and RNA polymerase II uses two different DNA basic strands as templates. The expression of RNA polymerase I and RNA polymerase II is designed to transcribe two different DNA basic strands, resulting in two complementary RNA strands. Thus, this structure ensures that both antisense RNA strands and righteous RNA strands are obtained from a single cDNA strand. Meanwhile, after the antisense RNA strand and the righteous RNA strand are expressed in the host cell, the righteous RNA starts to translate the viral protein as mRNA. Similar to the process of infection of cells by common viruses, virus assembly and cell lysis proceed sequentially [8].

Some viruses have genes that are segmented. In engineered bacteria, different gene fragments of these viruses must be imported into the plasmid to express the complete viral genome. It was shown that viral fragments can be automatically assembled after expression in engineered bacteria. In addition, each newly generated viral particle contains all fragment genes of the virus, which are not duplicated.

The virus was fully expressed in the engineered bacteria and could be detected from the cell culture after cell lysis. After cell pyrolysis, the highest virus concentration is in the supernatant. Therefore, a large number of viruses can be collected.

### 5.1. Viral Vector Vaccine

Viral vector vaccines are designed to amplify the COVID-19 antigen in the human body by feeding the viral antigen gene into a viral vector, thereby triggering an immune response to the COVID-19 antigen in the body. The virus usually used as a vector is generally called adenovirus, because adenovirus stimulates the body to produce strong humoral or cellular immunity. In addition, adenoviruses are highly capable of infecting the respiratory and intestinal tracts, causing rapid dispersion of infected cells and producing an even stronger immune response in the body. Adenoviruses offer several advantages and have become a more desirable solution for viral vector vaccines.

As a viral vector, adenovirus is a genetic mutant of the original adenovirus. Adenovirus can trigger a strong immune response in the body even after deletion of the E1 or E3 genes. Therefore, adenoviruses must be purified before they can be safely used. This virus is known as an i-generation virus. Due to the deletion of E2 or E4, the immune response to adenovirus infection is reduced and the viral genes are less packaged, but the safety is increased. This virus is known as “second generation.” When all or most of the adenovirus genes are deleted, the virus is called a third-generation virus and the immune response is very low. Considering the efficiency of the immune response, the first generation is often used as a vaccine vector, which accelerates the onset of the immune response.

In summary, the S protein of COVID-19 is strongly antigenic. Therefore, expression of the S protein of COVID-19 in vivo elicits an effective epitope response. The cDNA expressing the S protein was integrated into the genome of a generation of adenovirus. Isolated human respiratory cells were then infected with adenovirus, and the products of the infected cells were detected by western blot. The S protein was observed to be produced or not. The next experiment was started after the test.

### 5.2. Recombinant Protein Vaccine

According to the abovementioned analysis, the S protein is essential for the human body to produce an immune response to COVID-19. Recombinant protein vaccines are synthesized in large amounts, and the S protein is made into a vaccine that is injected into the human body. A large amount of S protein appears in the human body and is observed as an antigen by the immune system, resulting in the production of antibodies to S protein through the organism. This antibody can bind to COVID-19 at the same time and trigger an immune response.

The production of S protein is mainly dependent on the engineered bacteria. The mRNA required for the translation of the S protein can be obtained by sequencing and structural detection of the S protein. cDNA expressing the S protein is obtained from the mRNA, which is inserted into a plasmid to obtain a recombinant plasmid expressing the S protein. The recombinant plasmid was imported into the engineered bacteria such as *E. coli* and *Bacillus subtilis*. The S protein was detected by western blot, and the engineered bacteria that successfully expressed S protein were selected for further screening. The bacteria with high S protein expression can be screened by a directed evolution strategy and mass production of bacteria can be realized. Highly pure S proteins can be isolated and extracted from bacterial products for use as vaccines.

### 5.3. mRNA Vaccines

The mRNA binds directly to the ribosome inside the cell and translates the peptide chain. Messenger RNA vaccines are injected into receptors by selecting messenger RNA capable of translating viral antigenic proteins. Mass production of antigenic proteins is achieved through the receptor's synthesis mechanism, and antibodies specific for the antigenic protein are formed based on the immune system's response to the antigenic protein.

The mRNA for synthesizing antigenic proteins is not the only component of an mRNA vaccine. Due to the instability of RNA structure, RNA hydrolases are abundant in the living body and in the environment, making it impossible for ordinary RNA to survive stably in the living body for a long time. Therefore, the development of mRNA vaccines requires modification of mRNA to prolong its effectiveness in the environment. To prolong the life of mRNA, it is processed into non-self-amplifying mRNA and self-amplifying mRNA.

Self-amplifying mRNA vaccines: there is an arbovirus that belongs to the class A virus. It is an RNA virus that can replicate independently in the human body and produce a strong immune response. Structural genes and genes related to toxin expression can be knocked out by biotechnological means to maintain only its own replication function [9]. Subsequently, mRNAs that can translate S proteins are integrated into the RNA virus, giving the mRNA the ability to self-replicate.

Non-self-amplifying mRNA vaccine: this vaccine is mainly used to modify mRNA and increase the stability of mRNA in cells. Utr structure is added to the 5′ segment of mRNA. At the same time, the poly A tail is added to the 3′ segment. Such modified RNA is difficult to bind to RNA hydrolase and also prolongs the residence time of mRNA in the cell. Unlike self-amplifying mRNAs, non-self-amplifying mRNAs are not viruses and do not have the ability to self-infect and self-replicate. Therefore, non-self-amplified mRNA vaccines cannot enter cells directly and must be injected accurately into the recipient cells to produce the target S protein.

## 6. Conclusions and Prospects

The development of vaccines and specific drugs takes a long time, ranging from tens of months to 5 years. The theoretical concepts of synthetic biology are gaining popularity in a short period of time, but provide a very powerful motivation for research. Unlike traditional biomedicine, the concept of synthetic biology allows the integration of multiple disciplines and the multifaceted analysis of novel coronaviruses, which can significantly facilitate vaccine development. However, COVID-19 will coexist with humans for a considerable period of time in the foreseeable future. Until a vaccine is developed, humans can only reduce the chance of virus transmission through social appeals and executive orders.

## Data Availability

The datasets used and/or analyzed during the current study are available from the corresponding author on reasonable request.
